The article "A Review of Routine Laboratory Biomarkers for the Detection of Severe COVID-19 Disease" was published in 2022. Journal: Int J Anal Chem.

# A Review of Routine Laboratory Biomarkers for the Detection of Severe COVID-19 Disease

**DOI:** 10.1155/2022/9006487

**Published:** 2022-10-11

**Authors:** Keynaz Keykavousi, Fahimeh Nourbakhsh, Nooshin Abdollahpour, Farzaneh Fazeli, Alireza Sedaghat, Vahid Soheili, Amirhossein Sahebkar

**Affiliations:** ^1^Department of Pharmaceutical Control, School of Pharmacy, Mashhad University of Medical Sciences, Mashhad, Iran; ^2^Medical Toxicology Research Centre, Faculty of Medicine, Mashhad University of Medical Sciences, Mashhad, Iran; ^3^Department of Biology, Faculty of Sciences, Young Researchers and Elite Club, Islamic Azad University-Mashhad Branch, Mashhad, Iran; ^4^Department of Anesthesiology, Mashhad University of Medical Sciences, Mashhad, Iran; ^5^Lung Diseases Research Center, Faculty of Medicine, Mashhad University of Medical Sciences, Mashhad, Iran; ^6^Applied Biomedical Research Center, Mashhad University of Medical Sciences, Mashhad, Iran; ^7^Biotechnology Research Center, Pharmaceutical Technology Institute, Mashhad University of Medical Sciences, Mashhad, Iran; ^8^School of Medicine, The University of Western Australia, Perth, Australia

## Abstract

As the COVID-19 pandemic continues, there is an urgent need to identify clinical and laboratory predictors of disease severity and prognosis. Once the coronavirus enters the cell, it triggers additional events via different signaling pathways. Cellular and molecular deregulation evoked by coronavirus infection can manifest as changes in laboratory findings. Understanding the relationship between laboratory biomarkers and COVID-19 outcomes would help in developing a risk-stratified approach to the treatment of patients with this disease. The purpose of this review is to investigate the role of hematological (white blood cell (WBC), lymphocyte, and neutrophil count, neutrophil-to-lymphocyte ratio (NLR), platelet, and red blood cell (RBC) count), inflammatory (C-reactive protein (CRP), erythrocyte sedimentation rate (ESR), and lactate dehydrogenase (LDH)), and biochemical (Albumin, aspartate aminotransferase (AST) and alanine aminotransferase (ALT), blood urea nitrogen (BUN), creatinine, D-dimer, total Cholesterol, low-density lipoprotein (LDL), and high-density lipoprotein (HDL)) biomarkers in the pathogenesis of COVID-19 disease and how their levels vary according to disease severity.

## 1. Introduction

Since the onset of the new coronavirus (SARS-CoV-2 (severe acute respiratory syndrome coronavirus-2), previously known as 2019-nCoV) pandemic in December 2019 [1, 2], confirmed cases have been reported in countries all over the world. The World Health Organization proclaimed the 2019 coronavirus disease (COVID-19) pandemic on March 11, 2020, mostly because of the disease's pervasive development [3]. Prior to that, it began as an outbreak in mainland China, with the first reports coming from the city of Wuhan in the province of Hubei on February 26, 2020. After the virus' genome was sequenced, the virus was given the name severe acute respiratory syndrome coronavirus-2 (SARS-CoV-2) by the International Committee on Taxonomy of Viruses. It shared genetic ancestry with the coronavirus outbreak that caused the SARS epidemic of 2003 [4]. Until July 30, 2022, COVID-19, the disease caused by SARS-CoV-2 virus infection, has posed a very significant threat to global public health with a total of 581,182,629 reported cases and 6,418,043 mortalities documented [5]. With 3,987,543 cases, the American continent was among those with the largest number of cases, with the United States and Brazil as the leading countries (2,137,731 and 923,189, respectively) [5, 6].

The article "A Review of Routine Laboratory Biomarkers for the Detection of Severe COVID-19 Disease" was published in 2022. Journal: Int J Anal Chem.

SARS-CoV-2 virus belongs to the order Nidovirales, suborder Cornidovirineae, family Coronaviridae, and subfamily Orthocoronavirinae. SARS-CoV-2 is an enveloped and symmetrical virus with spike-like projections on its membrane, giving it the shape of crowns. It has a positive-sense single-stranded RNA genome (Figure 1) [7, 8].

The COVID-19 pathogenesis includes direct cytotoxicity of virus in ACE2 (angiotensin-converting enzyme 2)-expressing cells; Renin-Angiotensin-Aldosterone System (RAAS) dysregulation secondary to virus-mediated ACE2 downregulation; immune response dysregulation; damage to the endothelial cells and thromboinflammation; and tissue fibrosis (Figure 2) [9]. The heterogeneous course of COVID-19 disease is unpredictable, with most patients presenting with mild, self-limiting symptoms. The virus infection commonly starts with flu-like symptoms [10] and can be asymptomatic or may have a minor to severe development [11]. Despite this, up to 30% of patients require hospitalization, and up to 17% of them need intensive care support for acute respiratory distress syndrome (ARDS), hyper-inflammatory responses, and multiorgan failure [12, 13].

The predominant clinical symptoms, presented by individuals infected during the COVID-19 pandemic, are respiratory which is similar to the SARS and Middle East respiratory syndrome (MERS) outbreaks. Roughly 80% of infected people have mild to moderate symptoms. The remaining patients have severe disease that necessitates inpatient care [14]. The overall mortality rate seems to be around 3.8% [2, 15–18].

Fever (83%–98%), cough (50%–82%), fatigue (25%–44%), shortness of breath (19%–55%), and muscle soreness (11%–44%) have been reported to be the most common symptoms of COVID-19 infection. Other symptoms might include headache, sore throat, sputum production, rhinorrhea, chest tightness, nausea, vomiting, diarrhea, ageusia, and anosmia [15, 19].

The article "A Review of Routine Laboratory Biomarkers for the Detection of Severe COVID-19 Disease" was published in 2022. Journal: Int J Anal Chem.

A small percentage of infected people have no or moderate symptoms, whereas most of the cases have a severe or crucial prognosis, and some people die as a result. Although elderly patients with underlying conditions appear to be more vulnerable to serious sickness and death, there are incidences of life-threatening disease in healthy people. As a result, certain critical issues remained unresolved, as for why does illness intensity differ between individuals? How do some people have a more serious sickness than others? The variability of the COVID-19 clinical phenotype may be addressed by several parameters relating to the host, virus, and environment [20].

The interpretation and understanding of host variables, particularly genetic construction, has largely remained unclear. On the other hand, there is limited information on the pathophysiology of SARS-CoV-2 and only a few educated guesses about the virus' behavior. Scientists are just now starting to understand how host, viral, and environmental variables interplay to impact infection. In fact, people of any age, particularly older adults with comorbidities like chronic bronchitis [21], diabetes [22], hypertension [23], cardiovascular disease [24], lung and liver diseases [25], chronic kidney disease (CKD) [26], and chronic obstructive pulmonary disease (COPD) [21], may present with more severe disease. Furthermore, disorders and therapies that damage the immune system, including cancer therapy, bone marrow or organ transplantation, and long-term use of corticosteroids, may increase the risk of disease, leading to more serious prognosis, and even death [27, 28]. On the other hand, despite the fact that epidemiological data in some research found no indication of a greater transmission of SARS-CoV-2 among asthma patients, it appears that patients with nonallergic asthma had a more severe COVID-19 infection than patients with allergic asthma [29]. Importantly, during metabolic syndrome, the disease's deteriorated prognosis might be attributed to the three factors of this syndrome including hypertension, type 2 diabetes, and obesity, which are all risk factors for COVID-19 severity. Along with these well-known risk factors, there are other host-related variables that might influence COVID-19's result [20]. It has been shown in numerous studies, the SARS-CoV-2 virus affects not only the respiratory tract, but also other systems and organs such as the heart, liver, and gastrointestinal system. Some studies have shown that several important biochemical and hematological indicators are altered in COVID-19 patients [30–32]. These biomarkers may be useful for predicting prognosis and also for treatment management, especially in cases with comorbidities and/or a severe disease course [33].

The article "A Review of Routine Laboratory Biomarkers for the Detection of Severe COVID-19 Disease" was published in 2022. Journal: Int J Anal Chem.

According to studies, severe or fatal COVID-19 cases are associated with significantly increased white blood cell counts (WBCs), liver and kidney function markers, blood urea nitrogen (BUN), creatinine, C-reactive protein (CRP), lactate dehydrogenase (LDH), D-dimer, calprotectin, and interleukin-6 (IL-6). They are also associated with lower lymphocyte and platelet counts, as well as lower albumin levels, compared to milder cases in which the patients survived [34–38]. COVID-19 infection causes great burden of inflammation and neutrophil-to-lymphocyte ratio (NLR) is a novel marker of inflammation in certain conditions such as thyroid conditions [39], irritable bowel disease [40], and COVID-19 infection [41], cardiac conditions [42], and Hashimoto's disease [43].

Understanding the relationship between these biomarkers and COVID-19 outcomes would help in developing a risk-stratified approach to the treatment of patients with this disease. The purpose of this article is to investigate the role of hematological, inflammatory, and biochemical biomarkers in the pathogenesis of COVID-19 disease and how their levels vary according to the disease severity.

## 2. Biomarkers Associated with COVID-19 Infection and Severity

### 2.1. Hematological Biomarkers

One of the most commonly requested blood tests in clinical practice is the complete blood count (CBC) [44]. For too long, it has been used to quickly determine if a patient is anemic or infected, as well as to evaluate the blood's ability to coagulate normally [45].

White blood cell (WBC) count, lymphocyte count, neutrophil count, neutrophil-to-lymphocyte ratio (NLR), platelet count, and red blood cell (RBC) count are among the hematological biomarkers applied to stratify COVID-19 patients.

#### 2.1.1. WBC Count

In a study of 140 hospitalized COVID-19 patients confirmed by computed tomography (CT) scan findings, Zhang et al. found that the leukocyte count was within normal range in 68.1% of patients, decreased in 19.6% of them, and increased in 12.3% of them. They also observed that 75.4% of patients had lymphopenia [46]. On the other hand, Qin and colleagues investigated immune response dysregulation markers in 452 confirmed COVID-19 patients. They reported that severe cases had higher leukocyte counts [47]. In a meta-analysis of 21 studies involving 3377 COVID-19 positive patients, Henry et al. discovered that patients with serious and fatal disease had considerably higher WBC in comparison to nonsevere patients [48]. In a study conducted by Mardani et al., hematological biomarkers were compared between 70 COVID-19 positive patients and 130 COVID-19 negative patients. It has been investigated that RT-PCR positive group had significantly lower WBC counts than the negative control group [49].

The article "A Review of Routine Laboratory Biomarkers for the Detection of Severe COVID-19 Disease" was published in 2022. Journal: Int J Anal Chem.

In a retrospective cohort study of 219 COVID-19 patients, a higher white blood cell (WBC) count was linked to an increased risk of one-month mortality, according to the findings [50]. Moreover, Ferrari et al., in a retrospective study, reported that patients with COVID-19 had significantly higher WBC counts compared to controls [51]. Overall, the current evidence suggests that, while WBC count can be utilized as a predictive factor for severer COVID-19 conditions, the research findings are not consistent and further studies are required.

#### 2.1.2. Lymphocyte Count

Yang et al. [52] found lymphopenia in 80% of severely ill adult COVID-19 patients, while Chen et al. [15] found it in only 25% of mild infected patients. These findings suggest that lymphopenia may be related to the severity of infection. As observed by Henry et al., severe and fatal cases of COVID-19 tend to have a lower lymphocyte count than mild cases [48]. These findings were also confirmed by Qin et al. [47].

Chen et al. in a multicentric, retrospective study of 548 confirmed COVID-19 patients reported that survivors and nonsurvivors had significantly different hematological biomarkers on admission and at the end point. In fact, on admission, severe and critical cases, as well as nonsurvivors, had significant lymphopenia [53]. A meta-analysis of 20 publications found statistically significant decreases in total lymphocytes, CD4+ and CD8+ T-cells, and B-cells in critically ill COVID-19 patients compared to patients with moderate or mild disease [54]. Moutchia et al., in their systematic review, also reported that severe and critical cases of COVID-19 were characterized by lower lymphocyte and CD4 counts [55]. Due to the significant prevalence of lymphopenia in COVID-19 patients and its strong correlation with disease severity, current research suggests that lymphocyte count, particularly CD4+ levels, can be employed as a predictive biomarker for disease severity.

#### 2.1.3. Neutrophil Count

According to the available evidence, neutrophilia is an expression of a cytokine storm and hyperinflammatory state that play a key role in the pathogenesis of COVID-19 [2, 56]. Furthermore, neutrophilia can be caused by a secondary bacterial infection, which is more common in patients with advanced disease [14]. Chen and colleagues, in their study, observed that on admission, severe and critical cases, as well as nonsurvivors, had significantly increased neutrophil count compared with mild cases [53]. As reported by Mardani et al., confirmed COVID-19 patients have a significant increase in neutrophil count in comparison to the control group [49]. Moutchia et al., in a systematic review of 45 studies, observed that compared to nonsevere COVID-19 cases, patients with severe or critical COVID-19 have higher neutrophil counts [55]. In a retrospective cohort study of 201 COVID-19 patients, bivariate Cox regression analysis revealed that neutrophilia was linked to the development of acute respiratory distress syndrome (ARDS) and the progression from ARDS to death [57]. These studies demonstrated that neutrophilia in COVID‐19 patients was associated with the severity of the disease.

The article "A Review of Routine Laboratory Biomarkers for the Detection of Severe COVID-19 Disease" was published in 2022. Journal: Int J Anal Chem.

#### 2.1.4. Neutrophil-to-Lymphocyte Ratio (NLR)

Neutrophil-to-lymphocyte ratio (NLR) was first considered in the esophageal carcinoma patients under chemotherapeutic treatment, by dividing the relative percentage of neutrophils by lymphocytes. While the normal reference range in healthy population is 1–3, the values greater than 3 reveal an ongoing infection, and a ratio greater than 9 indicates sepsis. Therefore, the NLR value is associated with current inflammation as a prognostic biomarker [58].

As observed by Maet al., patients with a higher neutrophil-to-lymphocyte ratio (NLR>9.8) had a higher incidence of ARDS (*P* = 0.005), as well as higher rates of nonmechanical and mechanical ventilation (*P* = 0.002 and *P* = 0.048, respectively) [38]. Chen et al. also reported that in comparison to milder cases, severe and nonsurvivor COVID-19 cases had a higher neutrophil-to-lymphocyte ratio (NLR) as an inflammatory biomarker and a marker of systemic inflammation [53]. Qin and colleagues also published similar findings in their study [47]. In a retrospective, cross-sectional study, 101 COVID-19 positive patients were examined by means of hematological parameters. The ratio of neutrophils to lymphocytes showed a significant relationship with disease severity (*P* = 0.001) [59]. Moreover, as observed in a retrospective cohort study of 219 confirmed COVID-19 patients, a significant association between increased neutrophil-to-lymphocyte ratio (NLR) and increased risk of one-month mortality was reported [50]. Due to the relationship between increased neutrophil-to-lymphocyte ratio (NLR) and more severity of disease, NLR can be used as a prognostic marker in COVID-19 patients.

#### 2.1.5. Platelet Count

Platelet count has been suggested as a potential biomarker for COVID-19 patients, because it is a simple, inexpensive, and easily accessible biomarker which has been freely correlated with disease severity and mortality risk in the intensive care unit (ICU). Platelet count was found to be absolutely lower in COVID-19 patients [60], and it was lower in nonsurvivors in comparison to survivors [61]. Waris et al., in a retrospective cross-sectional study, found that the mean platelet count (165.0 × 10^9^/L) was significantly lower (*P* < 0.001) among critical COVID-19 patients compared to the mild group (217.0 × 10^9^/L) [59]. According to Chen et al., severe and nonsurvivor COVID-19 patients had significant thrombocytopenia, when compared to milder cases [53]. Henry et al., in their study, also discovered similar results and reported that patients with serious and fatal disease had significantly lower platelet counts in comparison to nonsevere patients [48].

The article "A Review of Routine Laboratory Biomarkers for the Detection of Severe COVID-19 Disease" was published in 2022. Journal: Int J Anal Chem.

Liu et al., in a retrospective study of 383 COVID-19 patients, reported that thrombocytopenia at the time of admission was linked to a nearly threefold increase in mortality rate compared to those who did not have thrombocytopenia. They also found that a 50 × 10^9^/L increase in platelet count was associated with a 40% reduction in mortality [62].

These studies demonstrated that lower platelet count in COVID‐19 cases was associated with disease severity.

#### 2.1.6. RBC Count

Liang et al. performed a study on the laboratory characteristics of 63 COVID-19 patients and investigated their efficacy for the diagnosis of the disease. They observed that, compared to healthy people, COVID-19 patients have lower levels of red blood cell (RBC) counts [11]. Taneri and colleagues conducted a systematic review to evaluate the biomarkers of anemia and iron metabolism. Compared with moderate COVID-19 patients, severe cases had a lower RBC count [63]. In a longitudinal cohort study of 379 COVID-19 patients, Lanini et al. reported that the mean RBC count was significantly lower in nonsurvivor patients compared to survivors. According to the temporal analysis, survivors and nonsurvivors had similar RBC counts at the time of symptom onset (*P*=0.257). The model predicted that by day 2 after the onset of symptoms, the average level of RBC would be significantly different between survivors and nonsurvivors [64]. The current evidence indicates that severe COVID-19 is associated with lower RBC counts in patients.

### 2.2. Inflammatory Biomarkers

According to the literature, C-reactive protein (CRP), erythrocyte sedimentation rate (ESR), and lactate dehydrogenase (LDH) are among the most prevalent inflammatory markers related to COVID-19 severity [65].

#### 2.2.1. CRP

C-reactive protein (CRP) is an acute-phase reactant generated by the liver and other organs in response to the release of IL-6, and it is a sensitive biomarker for a variety of inflammatory disorders like infection and tissue injury. Many patients with severe illness have high CRP levels [14]. In severe COVID-19 patients, the CRP marker was shown to be significantly elevated in the early stages of infection. It has also been linked to disease progression and is a predictor of severe COVID-19 [66]. In a retrospective cohort study of 140 confirmed COVID-19 patients, Liu et al. found that the proportion of patients with increased serum CRP levels was significantly higher among severe cases than in mild cases [67]. Another study investigated the association between CRP levels and lung lesions on CT scans. It was observed that, in the early stages of COVID-19, CRP levels were found to be strongly linked with the diameter of lung lesions and the severity of illness [68]. According to Stringer et al., a CRP level of 40 mg/L or above on admission to the hospital should be considered a reliable predictor of disease severity and increased mortality risk in COVID-19 patients [69]. Smilowitz et al., in their study, examined the relationship between serum CRP concentrations and adverse outcomes in hospitalized COVID-19 patients. The results suggested that CRP levels above the median (108 mg/L) were correlated with venous thromboembolism, acute kidney injury, critical illness, and mortality, in comparison with CRP levels below the median [70].

The article "A Review of Routine Laboratory Biomarkers for the Detection of Severe COVID-19 Disease" was published in 2022. Journal: Int J Anal Chem.

These studies suggest that CRP may be used for risk stratification of COVID-19 patients and early identification of disease severity, adverse outcomes, and mortality risk.

#### 2.2.2. ESR

The ESR is a measurement of the rate at which RBCs settle in a tube of anticoagulated blood over a given period. A wide range of immune and nonimmune factors can affect ESR, including changes in RBC quality and quantity, as well as changes in normal patterns and levels of different plasma proteins [71]. It has been demonstrated that severe COVID-19 is associated with a significant elevation in both ESR and CRP levels in the early stages of the disease. However, CRP changes are more sensitive to the disease condition [66]. Xiong and colleagues, in a study, analyzed the clinical, laboratory, and high-resolution CT scan findings of 42 COVID-19 patients. According to their results, the severity of pneumonia considered on the initial CT scan had a significant positive correlation with ESR. They suggested that an elevation in ESR, CRP, and LDH levels may be an indicator for the severity of inflammation or extensive tissue injury [72].

In a meta-analysis of 17 articles addressing inflammatory biomarkers in COVID-19 patients, Ghahramani et al. also confirmed the correlation between higher ESR levels and severity of the disease [73]. The available data indicate that due to the correlation between elevated ESR and higher disease severity, ESR can be used as a prognostic biomarker in COVID-19 patients.

The article "A Review of Routine Laboratory Biomarkers for the Detection of Severe COVID-19 Disease" was published in 2022. Journal: Int J Anal Chem.

#### 2.2.3. LDH

Lactate dehydrogenase (LDH) is an intracellular enzyme that catalyzes the oxidation of pyruvate to lactate during anaerobic glycolysis [74]. Serum LDH is routinely tested in clinical settings for a variety of diseases. Elevated serum LDH levels have been linked to a poor prognosis in a variety of diseases, particularly tumors and inflammation [56]. Despite the fact that LDH is an enzyme that originates from many organs, it increases significantly in patients with pulmonary involvement [75]. As noted by Wu et al., at the time of diagnosis, significant differences in serum LDH levels were detected between nonsevere and severe COVID-19 patients. It was also shown that an increase or decrease in LDH levels was a sign of radiographic improvement or progress [76]. Han et al., in a retrospective observational study of 107 confirmed COVID-19 patients, suggested that LDH has the potential to be identified as a powerful predictor for early detection of lung injury and severe cases [77]. According to a meta-analysis by Deng et al., 52% of COVID-19 patients had elevated LDH levels [31]. In a study of 123 hospitalized COVID-19 patients confirmed by RT-PCR, it was reported that serum LDH levels were elevated in 89% of patients. Another finding was the strong negative correlation between LDH and partial pressure of arterial oxygen to the fraction of inspired oxygen ratio (PaO_2_/FiO_2_) values, which is an indicator of patients' respiratory function. Therefore, it was concluded from this study that, to avoid a poor prognosis, LDH should be regarded as a useful test for the early identification of cases that need more aggressive supportive therapies and closer respiratory monitoring [78]. On the other hand, in a retrospective case-control study, Li et al. observed that an increased serum LDH level at admission is an independent risk factor for COVID-19 severity and mortality. They concluded that LDH can help with early COVID-19 detection [56]. Akdogan et al. reported that in the early stages of COVID-19, LDH levels were strongly linked to lung lesions, possibly reflecting disease severity [79].

From the current data, it can be concluded that an increased serum LDH level is linked to the severity of COVID-19 and it can be used for early detection of lung involvement, disease severity, and mortality risk.

#### 2.2.4. Inflammatory Cytokines

During SARS-CoV, MERS-CoV, and SARS-CoV-2 infection, scientists routinely focus on our current understanding of innate immune responses, inflammasome activation, inflammatory cell death pathways, and cytokines' release [80]. Cytokines are a type of polypeptide signaling molecule that acts on cell surface receptors to modulate a variety of biological activities [81]. Hyperproduction of mostly proinflammatory cytokines such as interleukin 1 (IL-1), IL-6, interleukin 12 (IL-12), interferon gamma (IFN-*ɣ*), and tumor necrosis factor alpha (TNF-*α*), which selectively target lung tissue, can significantly impair the prognosis in the most severe instances [82]. In critically sick COVD-19 patients, the cytokine storm can deteriorate the clinical symptoms or perhaps premature death. To enhance the survival rate of COVID-19 patients, early management of the cytokine storm using immunomodulatory and cytokine antagonists is critical.  Table1 offers the most important inflammatory factors during SARS-CoV-2 infection.

The article "A Review of Routine Laboratory Biomarkers for the Detection of Severe COVID-19 Disease" was published in 2022. Journal: Int J Anal Chem.

### 2.3. Biochemical Biomarkers

#### 2.3.1. Albumin

Albumin is a negative acute phase reactant with antioxidant properties. Therefore, under physiological circumstances, plasma albumin is a rich source of free thiols capable of scavenging reactive oxidant species. Under oxidative stress, albumin can undergo irreversible oxidation, impairing antioxidant properties and eventually causing cell and tissue damage [113]. In a systematic review and meta-analysis of 10 studies, in which a total of 1745 COVID-19 patients were evaluated, it was noted that 34% of patients demonstrated serum albumin levels lower than the normal range [31]. Wu et al. reported that at admission, the most common abnormal liver biochemical marker observed in COVID-19 cases was abnormal albumin [114]. In a recent article, Violi et al. investigated the predictive value of serum albumin for COVID-19 mortality. They observed that nonsurvivors had lower values of albumin in comparison to survivors. Cox regression analysis revealed that albumin was independently associated with mortality (hazard ratio: 2.48) after adjusting for sex, heart failure, chronic obstructive pulmonary disease (COPD), and CRP levels [113].

Li and colleagues found that lower levels of albumin were associated with increased severity of COVID-19 pneumonia. Even after adjusting for confounding factors, plasma albumin values in the critical group continued to have a significant correlation with the risk of mortality [76]. Due to the association between decreased serum albumin levels and higher disease severity, serum albumin can be used as a predictive biomarker for the severity of the disease in COVID-19 patients.

The article "A Review of Routine Laboratory Biomarkers for the Detection of Severe COVID-19 Disease" was published in 2022. Journal: Int J Anal Chem.

#### 2.3.2. AST & ALT

Abnormal liver function tests (LFTs) including elevated alanine aminotransferase (ALT) and aspartate aminotransferase (AST) are indicators of hepatocyte injury. However, it has been suggested that elevated aminotransferases in COVID-19 could also be caused by myositis rather than liver damage [115]. Deng et al., in their systematic review and meta-analysis, reported that ALT and aspartate AST values were found to be higher than normal in 16% and 20% of COVID-19 patients, respectively [31]. In a systematic review by Wu and colleagues, the incidence, risk factor, and prognosis of abnormal liver biomarkers in patients with COVID-19 were evaluated. They found that at admission, the pooled incidence of abnormal AST and ALT was 21.8% and 20.4%, respectively. Meta-analysis showed that serum AST and ALT levels were significantly increased in severe and critical cases compared to mild and moderate patients [114]. A recent systematic review and meta-analysis of 42 articles reported that, in nonsevere COVID-19 patients, an increase in ALT and AST levels was found in 30% and 21%, respectively, while in severe patients, it was found in 38% and 48% [116]. Canovi et al., in an observational cross-sectional study of 866 COVID-19 patients, observed that circulating concentrations of serum AST and ALT demonstrated a progressive increase with worsening parenchymal lesions [117]. The current evidence suggests that severe COVID-19 is correlated with higher AST and ALT levels in patients.

#### 2.3.3. Blood Urea Nitrogen (BUN)

Mudatsir et al., in a systematic review of 19 articles, observed that elevated levels of BUN were associated with severe COVID-19 [118]. Ghahramani et al., in their systematic review and meta-analysis, also reported that BUN levels showed a significant increase in severe patients compared to nonsevere ones [73]. In another meta-analysis, Danwang et al. confirmed this relation and discovered that severe COVID-19 patients tend to have higher levels of BUN [119]. Zhang and colleagues in a study of 289 COVID-19 patients observed that increased BUN on admission was found in survived severe cases compared to cases with nonsevere disease. They also reported high levels of this biomarker to be associated with in‐hospital death [120]. Moreover, as observed in a multicenter retrospective cohort study of 12,413 confirmed COVID-19 patients, a significant association between increased baseline BUN levels and increased risk of all-cause mortality was reported [121]. A recent study of 266 COVID-19 patients reported that compared with mild cases, severe patients had higher levels of BUN, proposing that BUN could be an independent element for predicting COVID-19 severity [122].

The article "A Review of Routine Laboratory Biomarkers for the Detection of Severe COVID-19 Disease" was published in 2022. Journal: Int J Anal Chem.

These studies showed that higher BUN concentrations in COVID‐19 cases were associated with higher disease severity and mortality rate.

#### 2.3.4. Serum Creatinine

As reported by Mudatsir et al., elevated levels of serum creatinine were correlated with severe manifestations of COVID-19 [118]. Ghahramani et al. also confirmed the association between higher creatinine levels and severity of disease in COVID 19-patients [73].

Danwang et al., in a meta-analysis, reported that serum creatinine levels are higher among COVID-19 severe cases in comparison to mild cases [119]. Zhang et al. confirmed that high levels of serum creatinine were associated with in-hospital mortality [120]. Liu et al. also observed that there was a relationship between elevated serum creatinine and increased all-cause mortality risk among COVID-19 cases [121]. Ferrando-vivas et al. in an observational cohort study of 10,362 critically ill patients discovered links between increased serum creatinine and higher 30-day mortality among COVID-19 cases, implying that deteriorating renal function was linked to a higher risk of death, as seen in many other types of critical illnesses [123]. Chen et al. in a study evaluated the impact of abnormal renal function on COVID-19 patients' prognosis and the prognostic value of various renal function indicators. They found that when adjusted for several important clinical variables, increased creatinine levels were independent predictors of mortality [124]. Current evidence suggests that serum creatinine can be used as a predictive biomarker for more severe COVID-19 cases and the risk of mortality.

#### 2.3.5. D-Dimer

The plasma cleavage product D-dimer is a breakdown product of cross-linked fibrin. During systemic fibrinolysis after alpha2 depletion, plasma may destroy fibrin monomers, cross-linked fibrin polymers, and perhaps fibrinogen [125]. A fibrin degradation product (FDP) refers to all of these fragments [126]. Although preventive anticoagulation in ICU patients in China was not widespread when these researches were conducted, increased D-dimer in COVID-19 patients has been linked to greater mortality in several publications. While the influence of anticoagulants on D-dimer levels, in the context of COVID-19, is unclear, individuals on anticoagulation therapy frequently have very low D-dimer levels [127]. However, it was demonstrated that there is a dynamic association between COVID-19 progression and the degree of D-dimer [128].

It was indicated that there is a relation between the asymptomatic deep vein thrombosis (DVT) and patients with pneumonia hospitalized due to the COVID-19 disease. Nevertheless, for the diagnosis of DVT in COVID-19 patients, higher D-dimer cut-off levels may be required [129]. Additionally, it was shown that D-dimer levels (above 2.0 g/mL) may reliably predict in-hospital mortality in COVID-19 patients. It is suggesting that D-dimer might be a helpful marker for better COVID-19 patient diagnosis [57, 130]. These results indicated that a higher D-dimer level in COVID-19 patients has been associated with an advanced death rate. Hence, D-dimer characterization can be one of the most valuable options for initial evaluation.

The article "A Review of Routine Laboratory Biomarkers for the Detection of Severe COVID-19 Disease" was published in 2022. Journal: Int J Anal Chem.

#### 2.3.6. Total Cholesterol

During a retrospective study including 597 hospitalized COVID-19 patients, Wei et al. reported that total cholesterol (TC) levels were significantly lower among COVID-19 cases in comparison to the control group [131]. In a meta-analysis of 22 studies, Zinellu et al. observed that total cholesterol (TC) levels were significantly lower in hospitalized COVID-19 patients with severe disease or nonsurvivor status [132]. Aparisi and colleagues, in a study, evaluated the correlation of lipid biomarkers with 30-days all-cause mortality among COVID-19 patients. They found that nonsurvivor cases had lower TC throughout the entire course of the disease [133]. Li et al. investigated the changes in lipid profile and their association with COVID-19 severity. They observed that TC levels showed an increasing trend in survivor cases, but showed a decreasing trend in nonsurvivor patients [120]. On the other hand, in a retrospective study, Qin et al. found that levels of total cholesterol were negatively correlated with length of hospital (LOS) stay in COVID-19 patients. They reported that at admission, serum levels of TC in the LOS >29 days group were significantly lower than those in the LOS ≤29 days group [134].

From the available literature, it can be stated that a lower total cholesterol (TC) level is linked to the severity of COVID-19, longer length of hospital (LOS) stay, and mortality risk.

#### 2.3.7. Low-Density Lipoprotein Cholesterol (LDL-c) and High-Density Lipoprotein Cholesterol (HDL-c)

In their study, Wei et al. reported that COVID-19 cases have significantly lower LDL-c levels in comparison to healthy subjects. Moreover, they reported that when compared to mild and severe cases, high-density lipoprotein cholesterol (HDL-c) levels only decreased significantly in critical cases [131]. According to Zinellu et al., patients with severe COVID-19 have significantly lower levels of HDL-c and LDL-c when compared to patients with milder disease [132]. As noted by Aparisi et al., nonsurvivor COVID-19 patients had lower LDL-c levels than survivors during their disease course [133]. According to Li et al., in severe COVID-19 patients, LDL-c and HDL-c tend to have increased levels in survivors compared with nonsurvivors [120]. Moreover, a cross-sectional retrospective study showed that COVID-19 patients had a serum HDL-c level of 1.02 ± 0.28 mmol/L, which was significantly lower compared to the control group (1.52 ± 0.55 mmol/L). Furthermore, the serum HDL-c quantity in the severe COVID-19 group was 0.83 ± 1.67 mmol/L, considerably lower than that in the other group, nonsevere COVID-19 patients (1.15 ± 0.27 mmol/L) [135]. On the other hand, Qin et al. in their study reported that the length of hospital stay was negatively correlated with serum HDL-c and LDL-c levels in COVID-19 patients. They found that serum HDL-c and LDL-c values were significantly lower in the LOS >29 days group compared to the LOS ≤29 days group at admission [134]. These studies indicate that the levels of serum HDL-c and LDL-c can be utilized for risk stratification of COVID-19 patients, identification of disease severity, length of hospitalization, and mortality risk. Common laboratory biomarkers and their relationship to the severity of COVID-19 are summarized in Table 2.

The article "A Review of Routine Laboratory Biomarkers for the Detection of Severe COVID-19 Disease" was published in 2022. Journal: Int J Anal Chem.

## 3. Conclusion

Since the beginning of COVID-19 outbreak, the capacity of hematological, biochemical, inflammatory, and immunological factors to predict patients with severe or fatal forms of COVID-19 has been of great scientific importance. To predict the severity of the disease in the early stages, it is critical to obtain a full profile of the laboratory analysis. According to the reviewed literature, hematological, inflammatory, and biochemical parameters are associated with severe prognosis in COVID-19 cases and can thus be used as predictive factors. This issue especially can be facilitated by evaluation of factors such as WBC, RBC platelet, lymphocyte, and neutrophil count, and NLR as hematological; CRP, ESR, and LDH as inflammatory; and Albumin, AST & ALT, BUN, creatinine, D-dimer, total Cholesterol, LDL, and HDL as biochemical biomarkers. However, it is important to know that the disease progression cannot be predicted by relying on only one or two factors, and it is crucial to monitor most of the elements together. On the other hand, while various possible therapeutic options for COVID-19 have been investigated, regulating proinflammatory responses to inactivate the virus could be the best treatment offer.

Thus, this review provided guidance for this prediction on hospital admission of patients to reduce the adverse effects of the disease. Such a prognosis could reduce unnecessary hospitalization of patients and the costs imposed on the health care system. Furthermore, these outcomes should be constantly re-evaluated according to the new findings, since more prospective cohorts with longer follow-up provided more useful and up-to-date data.

The article "A Review of Routine Laboratory Biomarkers for the Detection of Severe COVID-19 Disease" was published in 2022. Journal: Int J Anal Chem.

## Figures and Tables

**Figure 1:** Schematic structure of severe acute respiratory syndrome coronavirus-2 (SARS-CoV-2), an enveloped virus with single-stranded positive-sense (+sense) RNA taking four principal proteins, including membrane (M) and spike (S) glycoproteins, in addition to nucleocapsid (N) and envelope (E) proteins.

**Figure 2:** Mode of host entry and infective life cycle of severe acute respiratory syndrome coronavirus-2 (SARS-CoV-2) virus. **(1)** The interaction between the angiotensin-converting enzyme 2 (ACE2) receptor and S-protein leads to the attachment of the virus **(2)** The entry of virus conducted by endocytosis and/or by **(3)** Membrane fusion of virus **(4)** Translation of virus RNA leads to produce proteins 1a & 1ab **(5)** Proteolysis of proteins results in nonstructural proteins and replicase-transcriptase complex (RTC) **(6)** Synthesizing the new viral RNA (-sense) and the viral proteins **(7)** The association of the viral particle **(8)** Release of virus through exocytosis.

**Table 1:** The important inflammatory factors associated with COVID-19 infection.

Biomarker	Function	COVID‐19 cases	Outcome	Ref
**IL-1**	Main sources of monocyte activation	IL-1*β* can be activated and maturated during SARS-CoV-2	IL-1 shows an increase in viral load, mortality, lung damage, and loss of pulmonary function	[83, 84]
**IL-2**	IL-2 has an important role in the prevention of autoimmune diseases	Elevated levels of IL-2 have been observed in SARS-CoV-2	Elevated levels of IL-2 in patients with COVID-19	[85–87]
**IL-4**	It increases during activation and proliferation of B lymphocytes	Elevated IL-4 levels have been observed in SARS-CoV-2	IL-4 had negative effects on CD8^+^ memory T-cells during viral infection	[2, 15, 88]
**L-6**	IL-6 travels to the liver and induces a large number of acute-phase proteins such as (CRP), (SAA), and *α*_1_-antitrypsin	Elevated IL-6 levels have been observed in SARS-CoV-2	IL-6 induced cytokine storm	[89, 90]
**IL-7**	IL-7 has an important role in lymphocyte differentiation, peripheral homeostasis development of T-cells, and as a vaccine adjuvant	The role of IL-7 depends on IL-6 activity in SARS-CoV-2	IL-7 levels related to COVID-19 severity	[56, 91]
**IL-10**	Inhibits the production of proinflammatory cytokines	IL-10 can have immunostimulatory effects, such as stimulation of IFN-*γ* production by CD8^+^ T-cells	IL-10 levels increase in patients with COVID-19 than in those with MERS	[2, 92–94]
**IL-12**	IL-12 is one of a group of heterodimeric biomolecules with distinctive characteristics	IL-12 has key functions in the development of Th1 and Th17 cells, especially in SARS-CoV-2	Elevated serum IL-12 levels have been reported in patients infected with SARS-CoV-2	[15, 95–97]
**IL-13**	IL-13 is increased by activated Th2 cells	IL-13 has an important role in the development of bronchial asthma by increasing the production of TGF-*β*	There is association between the increase of IL-13 levels and the viral infection of SARS-CoV-2	[2, 98]
**IL-17**	IL-17 elevated in inflammatory processes and can be synthetized by Th17 lymphocytes	IL-17 is a proinflammatory cytokine with important role in tissue damage and infection	The Th17 cells can produce IL-17, which led to therapeutic approach for COVID-19 patients	[91, 99, 100]
**M-CSF**	M-CSF is the primary growth factor modulating the growth and development of hematopoietic lineage cells	Tyrosine-kinase III activated M-CSF, especially in SARS-CoV-2	M-CSF significantly elevated in patients with COVID-19 which is associated with lung damage and disease severity	[101, 102]
**G-CSF**	G-CSF is essential for the proliferation of polymorphonuclear granulocyte cells (PMNs)	Increased levels of G-CSF have been reported in SARS-CoV-2 infections and in patients with neutropenia	G-CSF levels directly related to the lung damage and viral load of SARS-CoV-2	[2, 57, 103, 104]
**IFN-*γ***	IFN-*γ* is a type-II IFN produced by a majority type of lymphocyte cells	IFN-*γ* participates in numerous immunological functions and in inflammatory processes such as SARS-CoV-2	IFN-*γ*, IL-6, and IL-10 levels were higher in patients with infection of SARS-CoV-2	[95, 105, 106]
**TNF-*α***	TNF-*α* is produced by various cell types, such as monocytes, macrophages, and T-cells	The serum TNF-*α* levels are significantly elevated in patients with COVID-19	TNF-*α* was one of the cytokines whose overproduction was related to a poor prognosis in patients with SARS-CoV-2	[106–111]
**VEGF**	VEGF is essential for vascular endothelial homeostasis and is present in numerous cells	VEGF hyper-regulation is observed in various viral infections, especially COVID-19	VEGF would be useful in the approach to the regeneration of lung tissue and treatment of lung fibrosis	[2, 107, 112]

The article "A Review of Routine Laboratory Biomarkers for the Detection of Severe COVID-19 Disease" was published in 2022. Journal: Int J Anal Chem.

**Table 2:** Biomarkers associated with the severity of COVID-19 infection.

	Biomarker	Normal range	COVID‐19 cases	Outcome	Ref
**Hematological biomarkers**	WBC count	4.5–11 × 10^3^ cells/mcL	Increase in WBC counts	WBC count can be utilized as a predictive factor for severe COVID-19 conditions	[46–51]
	Lymphocyte count	0.77–4.5 × 10^3^ cells/mcL	Lymphopenia, decreases in total lymphocytes, CD4^+^, CD8^+^ T-cells, and B-cells	Lymphocyte count, (particularly CD4+) levels, can be employed as a predictive biomarker	[52–55]
	Neutrophil count	0–1.2 × 10^3^ cells/mcL	Neutrophilia	Neutrophilia was linked to the development of ARDS	[14, 57]
	Neutrophil-to-lymphocyte ratio (NLR)	1–3	Increase in neutrophil-to-lymphocyte ratio	NLR can be used as a prognostic marker in COVID-19	[50, 53, 59]
	Platelet count	150–350 × 10^3^/mcL	Thrombocytopenia	Lower platelet count in COVID‐19 cases was associated with disease severity	[60–63]
	RBC count	20–30 mL/kg body weight	Decrease in RBC count	Severe COVID-19 is associated with lower RBC counts in patients	[63, 64]

**Inflammatory biomarkers**	CRP	<0.8 mg/dL	Increase in CRP	CRP levels above the median (108 mg/L) were correlated with venous thromboembolic disease, acute kidney injury, critical illness, and mortality	[66–70]
	ESR	Male: <50 years old ≤15 mm/hr Female: <50 years old ≤20 mm/hr	Increase in ESR	ESR can be used as a prognostic biomarker in COVID-19 patients	[71–73]
	LDH	60–160 U/L	Decrease in LDH	Increased serum LDH level is linked to the severity of COVID-19 and it can be used for early detection of lung involvement	[76–79]

**Biochemical biomarkers**	Albumin	3.5 g/dl to 5.4 g/dl.	Decrease in Albumin	Serum albumin can be used as a predictive biomarker for the severity of the disease	[76, 113, 114]
	AST & ALT	<35 U/L	Increase in AST & ALT	The severe COVID-19 is correlated with higher AST and ALT levels	[115–117]
	Blood urea nitrogen (BUN)	8–20 mg/dL	Increase in BUN	BUN could be an independent element for predicting COVID-19 severity	[119–122]
	Serum creatinine (CR)	Men: 0.7–1.2 mg/dL Women: 0.5–1.0 mg/dL	Increase in CR	The serum creatinine can be used as a predictive biomarker for more severe COVID-19 cases and the risk of mortality	[73, 118, 122–124]
	D-dimer	<250 ng/mL	Increase in D-dimer	DVT in patients hospitalized with COVID-19 pneumonia and increased D-dimer levels is similar to that reported in previous studies	[57, 126, 127, 129]
	Total cholesterol	150–199 mg/dL	Decrease in total cholesterol	Lower total cholesterol level is linked to the severity of COVID-19, longer length of hospital stay, and mortality risk	[120, 131–134]
	HDL-c LDL-c	>40 mg/dl < 100 mg/dL	Decrease in HDL-c LDL-c	HDL-c and LDL-c can be utilized for risk stratification of COVID-19 patients, identification of disease severity, length of hospitalization, and mortality risk.	[120, 133–135]
